The article "HO-1/PINK1 Regulated Mitochondrial Fusion/Fission to Inhibit Pyroptosis and Attenuate Septic Acute Kidney Injury" was retracted in 2024. Reasons: signs of a paper mill; suspected computer-generated content; unreliable results or conclusions; concerns about the data.

# HO-1/PINK1 Regulated Mitochondrial Fusion/Fission to Inhibit Pyroptosis and Attenuate Septic Acute Kidney Injury

**DOI:** 10.1155/2020/2148706

**Published:** 2020-10-22

**Authors:** Hai-Bo Li, Xi-Zhe Zhang, Yi Sun, Qi Zhou, Jian-Nan Song, Zhan-Fei Hu, Yun Li, Jian-Nan Wu, Ying Guo, Yuan Zhang, Jia Shi, Jian-Bo Yu

**Affiliations:** ^1^Department of Anesthesiology, Tianjin Medical University Nankai Hospital, Tianjin, China; ^2^Department of Anesthesiology, Chifeng Municipal Hospital, Inner Mongolia, China; ^3^Department of Anesthesiology, Tianjin Nankai Hospital, Tianjin, China

## Abstract

**Background:**

Endotoxin-associated acute kidney injury (AKI), a disease characterized by marked oxidative stress and inflammation disease, is a major cause of mortality in critically ill patients. Mitochondrial fission and pyroptosis often occur in AKI. However, the underlying biological pathways involved in endotoxin AKI remain poorly understood, especially those related to mitochondrial dynamics equilibrium disregulation and pyroptosis. Previous studies suggest that heme oxygenase- (HO-) 1 confers cytoprotection against AKI during endotoxic shock, and PTEN-induced putative kinase 1 (PINK1) takes part in mitochondrial dysfunction. Thus, in this study, we examine the roles of HO-1/PINK1 in maintaining the dynamic process of mitochondrial fusion/fission to inhibit pyroptosis and mitigate acute kidney injury in rats exposed to endotoxin.

**Methods:**

An endotoxin-associated AKI model induced by lipopolysaccharide (LPS) was used in our study. Wild-type (WT) rats and PINK1 knockout (PINK1KO) rats, respectively, were divided into four groups: the control, LPS, Znpp+LPS, and Hemin+LPS groups. Rats were sacrificed 6 h after intraperitoneal injecting LPS to assess renal function, oxidative stress, and inflammation by plasma. Mitochondrial dynamics, morphology, and pyroptosis were evaluated by histological examinations.

**Results:**

In the rats with LPS-induced endotoxemia, the expression of HO-1 and PINK1 were upregulated at both mRNA and protein levels. These rats also exhibited inflammatory response, oxidative stress, mitochondrial fission, pyroptosis, and decreased renal function. After upregulating HO-1 in normal rats, pyroptosis was inhibited; mitochondrial fission and inflammatory response to oxidative stress were decreased; and the renal function was improved. The effects were reversed by adding Znpp (a type of HO-1 inhibitor). Finally, after PINK1 knockout, there is no statistical difference in the LPS-treated group and Hemin or Znpp pretreated group.

**Conclusions:**

HO-1 inhibits inflammation response and oxidative stress and regulates mitochondria fusion/fission to inhibit pyroptosis, which can alleviate endotoxin-induced AKI by PINK1.

## 1. Introduction

Endotoxin is a common cause of morbidity and mortality of critically ill patients in clinical practice [1]. The most frequently infected organ by endotoxin is the kidney, whose infection usually results in endotoxin-associated acute kidney injury (AKI), a disease characterized by the rapid renal function decline [2]. The mortality of patients who suffer from AKI with sepsis is 30-60%, which is approximately twice of patients without AKI [3–5]. The pathophysiology of endotoxin-induced AKI is characterized by an overwhelming inflammatory response and oxidative stress that leads to tubular damage [6, 7].

Previous studies have shown that persistent inflammation and oxidative stress results in changes in the mitochondrial dynamics and the degradation process of injured mitochondrial in LPS-induced AKI [8, 9]. The correct morphology and effective function of the mitochondria are maintained through the dynamic balance of fusion/fission events, so that cells can actively and effectively adapt to environmental changes [10]. Early body subjected to stress, mitochondrial fission/fusion adaptive change, when excessive mitochondrial damage, mitochondrial fission than fusion, cause the cells death [8, 11, 12]. In cell death, mitochondrial fission precedes caspase activation and chromosome condensation. Pyroptosis is a form of inflammatory programed cell death pathway activated by human and mouse caspase1 and release of pro-inflammatory cytokines, including interleukin- (IL-) 1*β* [13]. Once activated, caspase1 cleaves pro-IL-1*β* into their mature forms, to induce pyroptosis [14]. Pyroptosis is involved in the death of renal tubular epithelial cells after exposure to microbial infection [15].

The heme oxygenase, which consists of inducible and constitutive isozymes (HO-1, HO-2), catalyze the rate-limiting step in the metabolic conversion of heme to the bile pigments (i.e., biliverdin and bilirubin) and thus constitute a major intracellular source of iron and carbon monoxide (CO). HO-1 and the subsequent metabolites of heme catabolism seem to play vital roles in regulating important biological responses, including inflammation, oxidative stress, and cell survival [16, 17]. In recent years, people have paid much more attention to the protection of heme oxygenase, and its protection was gradually confirmed in acute kidney injury [18, 19]. In a previous study, HO-1 protects the kidney during septic shock, which has been confirmed systematically [20]. HO-1 can regulate PINK1 to the antioxidant and anti-inflammatory activity effect in several neurodegenerative diseases [21]. In recent years, the vital role of PINK1 has been found in mitophagy resulting in the accumulation of damaged mitochondria or the lack of intracellular substances during mitochondrial homeostasis quality control and bioenergy metabolism disorders or cell death [22, 23]. Several evidences indicate a potential regulatory influence of the PINK1 on the mitochondrial dynamics equilibrium between fusion and fission reactions [24]. HO-1can improve LPS-induced AKI by inhibiting inflammation and oxidative stress; however, its underlying mechanisms remain unknown. In this study, we hypothesized that HO-1 inhibited inflammation response and oxidative stress and regulated mitochondria fusion/fission to inhibit pyroptosis, which alleviated endotoxin-induced AKI by PINK1.

## 2. Materials and Methods

### 2.1. Animals

Two-month-old male Sprague-Dawley rats (160 to 185 g) were provided by the Laboratory Animal Center of the Nankai Clinical Institution of Tianjin Medical University, Tianjin, China. Two-month-old PINK1 knockout (PINK1KO) rats (160 to 185 g) were purchased from Beijing Baiao Saitu Gene Biotechnology Co. Ltd., Beijing, China. Wild-type and knockout animals used in the experiments were age- and weight-matched littermates. Rats were caged individually at 30 to 70% humidity (23 to 25°C) and acclimatized to a 12 h light-dark cycle with access to food and water ad libitum.

All the care and experimental procedures of rats were approved by the Animal Ethical and Welfare Committee (AEWC) of Institute of Radiation Medicine Chinese Academy of Medical Sciences (no.IRM-DWLL-201907) and were performed in accordance with ARRIVE guidelines developed by the National Center for the Replacement, Refinement, and Reduction of Animals in Research.

### 2.2. Establishment of LPS-Induced AKI Model

Rats were fasted for 12 h but allowed free access to water before induction of anesthesia. The rats received an intraperitoneal injection of 20% urethane (1.5 g/kg) that kept them anesthetized throughout the experiment. Lipopolysaccharide (10 mg/kg, i.p.) reconstituted with 1 ml sterile sodium chloride, 0.9%, was applied to replicate the experimental model of endotoxin-induced AKI. The rats were pretreated intraperitoneally with 10 *μ*mol/kg Znpp (in 50 mM sodium bicarbonate) and 50 mg/kg hemin (dissolved in 0.1 M sodium hydroxide) 1 h before LPS injection [10, 25]. The blood samples were collected at 6 h after lipopolysaccharide administration, and then, the rats were euthanized. The kidney tissue was harvested, snap-frozen in liquid nitrogen, and stored at -70°C for analytical examinations. All experiments were carried out in a specific pathogen-free animal lab.

### 2.3. Biochemical Analysis

Plasma was prepared as described above. The plasma blood urea nitrogen (BUN), creatinine (CRE), superoxide dismutase (SOD) activity, and malondialdehyde (MDA) levels were measured using commercial kits (Nanjing Jiancheng Bioengineer Institute, Nanjing, China).

### 2.4. Enzyme-Linked Immunosorbent Assay

Inflammatory factors IL-6, TNF-*α*, and neutrophil gelatinase-associated lipocalin (NGAL) and kidney injury molecule 1(KIM-1) in rats plasma were determined using enzyme-linked immunosorbent assay (ELISA) kit, respectively (Cusabio Life Science, Wuhan, China). Experimental procedures in the provided instruction manuals were strictly followed.

### 2.5. Histopathology in LPS-Induced AKI

Rats left kidneys were harvested, and kidney tissues were fixed in 4% paraformaldehyde (pH = 7.4) overnight, dehydrated, embedded in paraffin, sectioned (4 *μ*m), and stained with H&E. The quantitative analysis of the renal tubular injury was scored according to the Paller scoring method [26]. The total score was the sum of all scores in the renal tubular lumen with higher scores representing more severe damage: dilatation or flatness of renal tubules (1 point); brush border injury (1 point); shedding of brush border (2 points); and cast (2 points), detached, or necrotic cells in the lumen of the tubule (1 point) by two pathologists.

### 2.6. TUNEL Assay Analysis in LPS-Induced AKI

Pyroptosis was detected by the TdT-mediated dUTP nick-end labeling (TUNEL) method according to In Situ Cell Death Detection Kit (Roche, USA) and DAB detection kit. Briefly, routine dewaxing and dehydration of paraffin-embedded sections were incubated with protease K (20 g/ml dissolved in Tris/HCl, pH 7.4~8.0) at room temperature. Sections were washed with PBS twice; the water around the sample was dried; 50 Ul of TUNEL reaction mixed solution was added; the water around the sample was dried; 50 Ul reformer-POD was added and then incubated. Hematoxylin restaining of the nucleus, sealing the piece, image analysis by Image-Pro Plus (Media Cybernetics, American) were done.

### 2.7. Quantitative Real-Time PCR Analysis

Total RNA was isolated from the rat right kidney tissues using a high-purity RNA kit (Roche, Germany) and was quantified by absorbance at 260 nm using a spectrophotometer. Then, 5 *μ*l total RNA was reverse-transcribed into complementary DNA by using a reverse transcriptase (Promega, USA). The resulting complementary DNA was subjected to reverse transcription PCR with SYBR Green Master Mix on an ABI PRISM 7000 Sequence Detector System (Applied Biosystems, USA). Polymerase chain reaction (PCR) was carried out under the following conditions: 95°C, 30 s (1 cycle); 95°C, 5 s, 60°C,20 s (40 cycles); and 95°C, 5 s, 60°C, 60 s (1 cycle). The primers used for the study are shown in Table 1. The relative expression of genes was normalized to that of *β*-actin. The threshold cycle (Ct) was obtained from triplicate samples and averaged. Calculations were based on the *ΔΔ*Ct method using the equation *R* (ratio) = 2^−ΔΔCt^.

### 2.8. Western Blot Analysis

The expression of HO-1, PINK1, Mfn1/2, OPA1, Drp1, Fis1, and *β*-actin in the rats' right kidney tissues was determined by Western blotting. The kidney tissue was lysed and clarified by centrifugation at 10,000 g for 10 min at 4°C. Equal amounts of soluble protein were subjected to 15% sodium dodecyl sulfate-polyacrylamide gel electrophoresis and transferred onto a polyvinylidene fluoride membrane (Bio-Rad, USA). Membranes were blocked with 5% nonfat powdered milk in Tris-buffered saline and Tween 20 (TBST) and incubated further at 4°C overnight with primary antibodies for HO-1 (1 : 500) (10701-1-AP), Mfn1 (1 : 800) (ab104274), Mfn2 (1 : 800) (ab56889), OPA1 (1 : 800) (ab157457), Fis1 (1 : 500) (10956-1-AP), Drp1 (1 : 500) (ab184247), PINK1 (1 : 600) (23274-1-AP), caspase1 (1 : 800) (22915-1-AP), IL-1*β* (1 : 1,000) (ab9722), and *β*-actin (1 : 1,000) (TA-09). After being washed three times with TBST, the blots were incubated with horseradish peroxidase–conjugated anti-rabbit immunoglobulin G (1 : 3,000) (ZB2301) at room temperature for 1 h. The area and integrated optical density of the bands were analyzed using Image-Pro Plus 6.0 software (Media Cybernetics, Rockville, MD).

### 2.9. Transmission Electron Microstropy Analysis of Mitochondrial Morphology

The kidney from WT and PINK1KO rats for electron microscopy as previously described [23]. The cortical area of the kidney was fixed with 2.5% glutaraldehyde (Sigma, USA). Fixed samples were stained with 1% osmium tetroxide in phosphate-buffered saline (PBS), followed by dehydration in ethanol, and embedded in the EPON-Araldite mixture resin. After polymerization of EPON, 70 nm thick sections on the LKB Nova ultramicrotome (Stockholm, Sweden) were prepared. Sections were collected on a carbon-coated Cu grid and stained with a lead citrate; the stained sections were viewed by the electron microscope JEM-1400 (“JEOL,” Tokyo, Japan) at low magnification (×10,000) to reveal the mitochondria. The lengths of individual mitochondria were measured by tracing using NIH ImageJ software. For each cell, approximately 15 mitochondria in a representative area were measured. Less than 1% long (>2 *μ*m) mitochondria indicate the degree of mitochondrial fragmentation.

### 2.10. Statistical Analysis

The data were expressed as means ± SEM and analyzed with SPSS 23.0 statistical software. A one-way analysis of variance (ANOVA) followed by Tukey's post hoc test was used for multigroup comparison. The graphical analyses were performed using Prism 8.3.0 software (GraphPad, San Diego, Calif). *p* < 0.05 was considered statistically significant.

## 3. Results

### 3.1. The Relationship of HO-1 and PINK1 in LPS-Induced AKI

To prove the relationship between HO-1 and PINK1 in endotoxin AKI, we examined the expression of HO-1 and PINK1 in LPS-induced AKI (see Figure 1). The expression of HO-1 and PINK1 proteins and mRNA was increased when WT rats were treated with LPS. The expression of HO-1 and PINK1 proteins and mRNA was downregulated in HO-1 inhibitor (Znpp) pretreatment. The expression of HO-1 and PINK1 proteins and mRNA was upregulated in HO-1 promotor (Hemin) pretreatment. The expression of PINK1 proteins and mRNA is nearly not the expression in PINK1KO rats. There are no significantly different PINK1 expression in LPS, Znpp, and Hemin pretreatment in PINK1KO rats.

### 3.2. HO-1/PINK1 Pathway-Mediated Renal Function of Rats with LPS-Induced AKI

The degree of organ dysfunction induced by endotoxin is closely related to the mortality rate, and even a modest degree of organ dysfunction results in 10% mortality in patients hospitalized with infection. In this study, renal function was assessed in endotoxin rats. To estimate the mediated renal function effects of HO-1/PINK1, the levels of plasma creatinine (CRE), blood urea nitrogen (BUN), neutrophil gelatinase-associated lipocalin (NGAL), and kidney injury molecule 1 (KIM-1) were detected as shown in Figure 2. Under control condition, PINK1KO and WT rats showed similarly low levels of CRE, BUN, NGAL, and KIM-1, indicating that the PINK1KO rats have normal renal function. As expected, increased BUN, CRE, KIM-1, and NGAL levels were observed in the LPS group, compared with the control group; interestingly, Znpp pretreatment markedly increased the levels of BUN, CRE, KIM-1, and NGAL in the Znpp+LPS group of WT rats, compared with the LPS group. However, Hemin pretreatment markedly decreased the levels of BUN, CRE, KIM-1, and NGAL in the Hemin+LPS group of WT rats, which indicated the HO-1 protective renal function of rats with LPS-induced AKI. In addition, the above HO-1 protective effects disappeared in PINK1KO rats, the levels of BUN, CRE, KIM-1, and NGAL in the Znpp+LPS group and Hemin+LPS group is not significantly different, compared with the LPS group in PINK1KO rats, which indicated that HO-1 participated in the effects alleviating LPS-induced renal function decrease in the kidney by PINK1.

### 3.3. HO-1/PINK1 Pathway-Alleviated LPS-Induced Pathological Damage in the Kidney

To estimate the alleviated pathological damage effects of HO-1/PINK1, the tubular morphology of the kidney was detected as shown in Figure 3(a). As expected, the results showed that renal cast and detached cells were scattered in the renal tubular lumen together with vacuolar degeneration increased in the LPS-exposed group, including loss of brush border, formation of tubular casts, and sloughing of cells into the tubular lumen, compared with the control group. In detail, less renal cast and detached cells were scattered in the renal tubular lumen together with vacuolar degeneration increase in the Hemin+LPS group. Conversely, more renal cast and detached cells were scattered in the renal tubular lumen together with vacuolar degeneration increased in Znpp+LPS group. However, renal cast and detached cells scattered in the renal tubular lumen together with vacuolar degeneration in the Znpp+LPS group and Hemin+LPS group have no significant difference, compared with the LPS group in PINK1KO rats. To estimate the alleviated pathological damage effects of HO-1/PINK1, the tubular injury score of kidney was detected as shown in Figure 3(b). As expected, the tubular score increased in the LPS-exposed group, compared with the control group; Hemin pretreatment resulted in a decrease of the tubular score in the Hemin+LPS group and a decrease of the tubular score by Znpp pretreatment in the Znpp+LPS group, respectively, compared with the LPS group in WT rats. Conversely, the tubular score was increased in PINK1KO rats, compared with the WT rats after being exposed to LPS. In addition, the tubular score in the Znpp+LPS and Hemin+LPS groups has no significant difference, compared with the LPS group in PINK1KO rats. Collectively, these data indicated that the HO-1 participated in the effects alleviating LPS-induced pathological damage in the kidney by PINK1.

### 3.4. HO-1/PINK1 Pathway-Alleviated Inflammation and Oxidative Stress of the Kidney with LPS-Induced AKI

The occurrence and development of endotoxin AKI mainly result from excessive inflammatory cytokine release and oxidative stress. To estimate the anti-inflammation and antioxidative effects of HO-1/PINK1, the levels of IL-6, TNF-*α*, MDA, and SOD in the kidney were detected as shown in Figure 4. As shown in Figures 4(a) and 4(b), the results demonstrated that inflammation contents IL-6 and TNF-*α* were increased in the LPS group, compared with the control group. In detail, Znpp pretreatment inflammation contents IL-6 and TNF-*α* were increased in the Znpp+LPS group and IL-6 and TNF-*α* were decreased in the Hemin+LPS group, compared with the LPS group in WT rats. Conversely, the IL-6 and TNF-*α* were increased in PINK1KO rats, compared with the WT rats after being exposed to LPS. In addition, IL-6 and TNF-*α* in the Znpp+LPS and Hemin+LPS groups have no significant difference, compared with the LPS group in PINK1KO rats. As shown in Figures 4(c) and 4(d), the results demonstrated that oxidative stress contents MDA was increased and SOD was decreased in the LPS group, compared with the control group. In detail, Znpp pretreatment oxidative stress contents MDA was increased and SOD were decreased in Znpp+LPS group, conversely, in the Hemin+LPS group, compared with the LPS group in WT rats. In addition, MDA was increased and SOD was decreased in PINK1KO rats, compared with WT rats after being exposed to LPS. In addition, MDA and SOD in the Znpp+LPS group and Hemin+LPS group have no significant difference, compared with the LPS group in PINK1KO rats. Taken together, these data indicated that HO-1 participated in the effects alleviating LPS-induced inflammation and oxidative stress in the kidney by PINK1.

### 3.5. HO-1/PINK1 Pathway-Mediated Mitochondrial Dynamics in LPS-Induced AKI

To examine the effects of HO-1/PINK1 on mitochondrial dynamics, the several proven mitochondrial fusion (Mfn1/2, OPA1) and fission (Drp1, Fis1) proteins and mRNA were detected as shown in Figure 5. As expected, the expression of mitochondrial fission marker Drp1 and Fis1 proteins and mRNA was increased, and mitochondrial fusion marker Mfn1, Mfn2, and OPA1 proteins and mRNA were decreased in the LPS-exposed group compared with the control group in WT rats. Znpp pretreatment results in the levels of Mfn1, Mfn2, and OPA1 proteins and mRNA being decreased; the levels of Drp1 and Fis1 proteins and mRNA were increased in the Znpp+LPS group; Hemin pretreatment results in the levels of Mfn1, Mfn2, and OPA1 proteins and mRNA being increased; the levels of Drp1 and Fis1 proteins and mRNA were decreased in the Hemin+LPS group, compared with the LPS group in WT rats. However, the levels of Mfn1, Mfn2, OPA1, Drp1, and Fis1 proteins and mRNA were not significantly different in the Znpp+LPS group and Hemin+LPS group, compared with the LPS group in PINK1KO rats. Taken together, these data indicated that the HO-1 participated in the effects alleviating LPS-induced mitochondrial fission in the kidney by PINK1.

### 3.6. HO-1/PINK1 Pathway-Mediated Change in the Ultrastructure of Mitochondria in LPS-Induced AKI

Mitochondria dynamics equilibrium defines the balance of mitochondria fusion and fission. We examined mitochondria morphology in renal tubular cells of WT and PINK1KO rats by electron microscopy and morphometric analysis as described (Figure 6). As shown in Figure 6(a), the mitochondria in renal tubular cells of PINK1KO and WT rats were found to be similar in size and shape, with most mitochondria displaying a tubular structure with a length greater than 2 *μ*m. Many small and round, fragmentation, swelling, vacuoles in the mitochondrial matrix, and loss of cristae mitochondria with a length less than 2 *μ*m were observed in tubular cells that are LPS exposed indicating mitochondrial fragmentation, compared with the control group. In Znpp pretreatment, there are more small and round, fragmentation, swelling, vacuoles in the mitochondrial matrix, and loss of cristae mitochondria in the Znpp+LPS group, less fission mitochondria in the Hemin+LPS group, compared with the LPS group in WT rats. However, small and round, fragmentation, swelling, vacuoles in the mitochondrial matrix, and loss of cristae mitochondria in the Znpp+LPS group and Hemin+LPS group have no significant difference, compared with the LPS group in PINK1KO rats. For quantification, we counted the ratio of proximal tubule cell fragmented mitochondria (Figure 6(b)). As expected, the ratio of proximal tubule cell fragmented mitochondria increased in the LPS-exposed group, compared with the control group; Hemin pretreatment resulted in a decrease of the ratio of proximal tubule cell fragmented mitochondria in the Hemin+LPS group and an increase of the ratio of proximal tubule cell fragmented mitochondria by Znpp pretreatment in the Znpp+LPS group, respectively, compared with the LPS group in WT rats. Conversely, the ratio of proximal tubule cell fragmented mitochondria was increased in PINK1KO rats, compared with WT rats after being exposed LPS. In addition, the ratio of proximal tubule cell fragmented mitochondria in the Znpp+LPS and Hemin+LPS groups has no significant difference, compared with the LPS group in PINK1KO rats. Collectively, these data indicated that HO-1 participated in the effects alleviating LPS-induced mitochondrial morphology in the kidney by PINK1.

### 3.7. HO-1/PINK1 Pathway-Alleviated LPS-Induced Pyroptosis in Kidney

We further evaluated renal tubular cell pyroptosis by TUNEL assay as shown in Figure 7. As shown in Figures 7(a) and 7(b), cell swelling and lytic cell death were found in the LPS-exposed group; Znpp pretreatment results in more cell swelling, lytic cell death, and percentage of pyroptosis cells in the Znpp+LPS group, Hemin pretreatment results in less cell swelling, lytic cell death, and percentage of pyroptosis cells in the Hemin+LPS group, compared with the LPS group in WT rats. However, cell swelling, lytic cell death, and percentage of pyroptosis cells were not significantly different in the Znpp+LPS group and Hemin+LPS group, compared with the LPS group in PINK1KO rats. Additionally, consistent with the results of TUNEL assay, the expression of caspase1 and IL-1*β* protein and mRNA were revealed to be significantly increased in the LPS-exposed group, compared with the control group as shown in Figures 7(c) and 7(d). Hemin pretreatment resulted in a decrease of caspase1 and IL-1*β* proteins and mRNA; conversely, the expression of caspase1 and IL-1*β* proteins and mRNA were increased in Znpp pretreatment, compared with the LPS group in WT rats, which indicated that HO-1 inhibit the expression of caspase1 and IL-1*β*. The expression of caspase1 and IL-1*β* increased in PINK1KO rats than WT rats after LPS treatment. Additionally, there is significant difference among the LPS, Znpp+LPS, and Hemin+LPS groups in PINK1KO rats. Taken together, these data indicated that HO-1 participated in the effects alleviating LPS-induced pyroptosis in the kidney by PINK1.

## 4. Discussion

In the present study, our results demonstrated that underlying LPS induced AKI by focusing on inflammation response, oxidative stress, mitochondrial fission, and pyroptosis. HO-1 inhibited inflammation response and oxidative stress and regulated mitochondria fusion/fission to inhibited pyroptosis, which alleviated endotoxin-induced AKI by PINK1.

LPS, a known toxic component of Gram-negative bacteria [27], is used to induce AKI by intraperitoneal administration [28, 29]. In this study, the 6-hour time point was chosen after LPS treatment according to our previous study [20]. To clarify the effect of HO-1 on the kidney during endotoxemia, we administered Znpp and Hemin to rats according our previous study [20, 25]. After LPS treatment, the indicators of kidney injury (BUN, CRE, KIM-1, and NGAL) are significantly increased, the integrity of tubular structures is disrupted, and edema of renal tubular epithelial cells, tubular necrosis, and cast formation are observed, which suggest renal dysfunction and kidney injury. Oxidative stress and inflammation are known as the main pathological mechanisms of AKI [30]. LPS-induced AKI is coupled to oxidative stress biomarkers including MDA and SOD [30, 31]. LPS-induced AKI is coupled to higher levels of inflammatory cytokines including IL-6 and TNF-*α* [32]. Our results show that oxidative stress and inflammation occur in the kidney after the administration of LPS by analysis of SOD, MDA, IL-6, and TNF-*α*.

Oxidative stress and inflammation that occur in the kidney can induce mitochondria dynamic injury after being exposed to endotoxin. Mitochondrial dynamic include fusion and fission, which was a balance in the normal physiology. A mitochondrion fusion relies on mitofusin 1 (Mfn1) and mitofusion 2 (Mfn2) at the mitochondrial outer membrane and optic atrophy1 (OPA1) on the inner membrane, whereas fission relies on dynamin-related protein 1 (Drp1) translocation into the mitochondria to initiate fission by forming a spiral constriction ring with local receptors such as fission protein 1 (Fis1) on the outer membrane [33, 34]. However, the balance was skewed to favor fission in the endotoxin-induced AKI [33–35]. Changes in mitochondrial morphology, characterized by initial fragmentation of the organelles followed by ultrastructural alterations resulting in mitochondrial swelling and cristae deformation, are observed in renal tubular cells during septic AKI [8]. Our results show the mitochondrial swelling and cristae deformation in renal tubular cells, the expression of fusion includes Mfn1, Mfn2, and OPA1 proteins and mRNA upregulation, and the fission includes Drp1 and Fis1 proteins and mRNA downregulation in LPS-induced AKI.

Mitochondrial quality control is a key determinant of cell survival. Mitochondria are the energy-producing dynamic double-membrane organelles essential for cellular survival [36]. Programmed cell death is a defense against infection [14]. In cell death, mitochondrial fission precedes caspase activation and chromosome condensation. In the early stages of apoptosis initiation, Drp1 colocalizes Mfn2 at the OMM, forming a complex, which was hypothesized to prevent mitochondrial OMM fusion due to Mfn2 inhibition [37]. Drp1 localization to OMM is also responsible for mitochondrial fission for Drp1depletion or inhibition by expression of a dominant negative mutant (DrpK38A) preventing mitochondrial fragmentation, cyt c release, caspase activation, and apoptosis [38]. There are few studies on mitochondria involvement in pyroptosis in septic kidney injury, and the mechanism is not fully understood. Pyroptosis is a recently identified pathway of host cell death that is stimulated by a range of microbial infections and noninfectious stimuli. Pyroptosis is a form of inflammatory programed cell death pathway activated by human and mouse caspase1 and release of proinflammatory cytokines, including interleukin- (IL-) 1*β* [39]. Pyroptotic cell death has been confirmed in LPS-induced AKI [15]. Our results show that mitochondria fission precedes caspase1 and IL-1*β* activation involved pyroptosis occur in LPS-induced AKI.

Heme oxygenase-1 (HO-1) is a speed-limiting enzyme that catalyzes the degradation of heme into carbon monoxide (CO), bilirubin, and Fe^2+^. It is distributed in almost all tissues, playing an important regulatory role in a variety of physiological and pathological processes. A previous study has confirmed that HO-1 can alleviate AKI by inducing LPS [20]. Our results show that renal dysfunction and kidney injury increased in HO-1 inhibitor Znpp pretreatment, conversely, decreased in Hemin pretreatment. It is consistent with our previous study. Tissue and organ protection is exerted through multiple mechanisms such as antioxidation, anti-inflammation, and antiapoptosis [16, 40, 41]. Our results show that oxidative stress and inflammation decreased, mitochondrial fusion protein increased, fission protein decreased, and pyroptosis and the expression of caspase1 and IL-1*β* decreased by upregulated HO-1. Above, we confirm that HO-1 treatment, accompanied by inhibit inflammation, oxidative stress, and mitochondria fission, remarkably improved the AKI of endotoxin rats induced by LPS, which was associated with alleviated pyroptosis.

HO-1 can regulate PINK1 to antioxidant and anti-inflammatory activities effect in several neurodegenerative diseases [21]. PINK1 is widely expressed in the cells of the body, including the kidney, mainly in the mitochondrial intima. Several lines of evidence indicate a potential regulatory influence of the PINK1 on the mitochondrial dynamics equilibrium between fusion and fission reactions [24, 42]. During the cellular stress, PINK1 regulates the mitochondrial kinetic process and mediates the autophagic clearance of the mitochondria damaged by kidney injury [22, 23, 43]. Our results show that the levels of PINK1 proteins dramatically decreased by downregulated HO-1 in LPS-induced AKI, accompanied by inflammation, oxidative stress, mitochondria fission, and pyroptosis increase. Conversely, the levels of PINK1 increased by upregulated HO-1 in LPS-induced AKI, accompanied by inflammation, oxidative stress, mitochondria fission, and pyroptosis decrease. However, HO-1 cannot inhibit inflammation, oxidative stress, mitochondria fission, and pyroptosis during PINK1 knockout. These illustrated HO-1-inhibited inflammation, oxidative stress, mitochondria fission, and pyroptosis attenuate AKI-exposed endotoxin by PINK1.

There are several limitations in this study. First, we observed AKI only 6 h after LPS treatment, which still needs more time points to be explored further. Second, the mortality of endotoxin needs to be exhibited. Third, we observed only renal tubular cell mitochondria and pyroptosis in vivo; the effects of HO-1/PINK1 on renal tubular cell mitochondria and pyroptosis in vitro are required to investigate. Fourth, we observed the mitochondria fusion/fission biomarker and morphology, but the mitochondria function need is detected. Fifth, the mitochondria fission inhibiting pyroptosis need is investigated by using the mitochondria fission inhibitor. Collectively, more studies are required to investigate the mechanism of HO-1/PINK1 on endotoxin-induced AKI.

In conclusion, HO-1 inhibited inflammation response and oxidative stress and regulated mitochondria fusion/fission to inhibited pyroptosis, which alleviated endotoxin-induced AKI by PINK1.

## Figures and Tables

**Figure 1:** The relationship of HO-1/PINK1 protects against LPS-induced kidney injury. Representative immunoblot analysis of (a) HO-1 and (b) PINK1 in kidney tissues. Real-time PCR shows the relative expression of (c) HO-1 mRNA and (d) PINK1 mRNA in kidney tissues. Data are expressed as mean ± SEM, *n* = 6. ^∗^*p* < 0.05 versus the WT control group, ^#^*p* < 0.05 versus the WT LPS group, and ^&^*p* < 0.05 versus the PINK1KO LPS group. HO-1: heme oxygenase-1; PINK1: PTEN-induced putative kinase 1; LPS: lipopolysaccharide; Znpp: zinc protoporphyrin IX.

**Figure 2:** HO-1/PINK1 pathway-mediated renal function of rats with LPS-induced AKI. Levels of plasma BUN (a), CRE (b), KIM-1 (c), and NGAL (d). Data are expressed as mean ± SEM, *n* = 6, ^∗^*p* < 0.05 versus the WT control group, ^#^p < 0.05 versus the WT LPS group. WT: wild type; PINK1KO: PTEN-induced putative kinase 1 knockout; LPS: lipopolysaccharide; Znpp: zinc protoporphyrin IX; CRE: creatinine; BUN: blood urea nitrogen; KIM-1: kidney injury molecule-1; NGAL: neutrophil gelatinase-associated lipocalin.

**Figure 3:** HO-1/PINK1 alleviated LPS-induced pathological damage in the kidney. (a) The representative sections (hematoxylin and eosin (H & E) staining) of the rats' kidney. Original magnification, ×200; scale bar: 100 *μ*m. Pathological score of tubular damage (b). Data are expressed as mean ± SEM, *n* = 6, ^∗^*p* < 0.05 versus the WT control group, ^#^*p* < 0.05 versus the WT LPS group. WT: wild type; PINK1KO: PTEN-induced putative kinase 1 knockout; LPS: lipopolysaccharide, Znpp: zinc protoporphyrin IX.

**Figure 4:** HO-1/PINK1 pathway-alleviated inflammation and oxidative stress of kidney with LPS-induced AKI. Levels of plasma inflammation biomarker IL-6 (a) and TNF-*α* (b). Levels of plasma oxidative stress biomarker of MDA (c) and SOD (d). Data are expressed as mean ± SEM, *n* = 6, ^∗^*p* < 0.05 versus the WT control group, ^#^*p* < 0.05 versus the WT LPS group. WT: wild type; PINK1KO: PTEN-induced putative kinase 1 knockout; LPS: lipopolysaccharide; Znpp: zinc protoporphyrin IX; MDA: malondialdehyde; SOD: superoxide dismutase.

**Figure 5:** HO-1/PINK1-regulated mitochondrial dynamics. (a) Representative immunoblot analysis of (A) Mfn1, (B) Mfn2, (C) OPA1, (D) Drp1, and (E) Fis1 from kidney tissues. (b) Real-time PCR shows the relative expression of (A) Mfn1 mRNA, (B) Mfn2 mRNA, (C) OPA1 mRNA, (D) Drp1 mRNA, and (E) Fis1 mRNA from kidney tissues. Data are expressed as mean ± SEM, *n* = 6. ^∗^*p* < 0.05 versus the WT control group, ^#^*p* < 0.05 versus the WT LPS group. PINK1KO: PTEN-induced putative kinase 1 knockout; LPS, lipopolysaccharide; Znpp: zinc protoporphyrin IX; Mfn1: mitofusin 1; Mfn2: mitofusin 2; OPA1: optic atrophy 1; Drp1: dynamin-related protein 1; Fis1: mitochondrial fission 1.

**Figure 6:** HO-1/PINK1-regulated mitochondrial ultrastructure. (a) Representative transmission electron micrographs of the mitochondrial ultrastructure of kidney tissues. Scale bars: 2 *μ*m and 5 *μ*m. (b) Ratio of cell with fragmented mitochondria. Data are expressed as mean ± SEM, *n* = 3. ^∗^*p* < 0.05 versus the WT control group, ^#^*p* < 0.05 versus the WT LPS group. WT: wild type; PINK1KO: PTEN-induced putative kinase 1 knockout; LPS: lipopolysaccharide; Znpp: zinc protoporphyrin IX.

**Figure 7:** HO-1/PINK1 pathway-alleviated LPS-induced pyroptosis in kidney. (a) Representative images of TUNEL staining. Scale bar: 100 *μ*m. (b) Percentage of pyroptosis cells of tubular damage. (c) Western blot show the expression of caspase1 and IL-1*β* protein in kidney tissues of rats (A–C). (d) Real-time PCR shows the relative expression of (a) caspase1 mRNA and (b) IL-1*β* mRNA. Data are expressed as mean ± SEM, *n* = 6. ^∗^*p* < 0.05 versus the WT control group, ^#^*p* < 0.05 versus the WT LPS group. PINK1KO: PTEN-induced putative kinase 1 knockout; LPS: lipopolysaccharide; Znpp: zinc protoporphyrin IX.

**Table 1:** The primers used for the study.

Gene	Forward	Reverse
*HO-1*	5′ -GAC AGA GTT TCT TCG CCA GA -3′	5′ -GCC ACG GTC GCC AAC AGG AA-3′
*PINK1*	5′- CTA CCG CTT CTT CCG CCA GTC -3′	5′- CCG CCT GCT TCT CCT CGA TCA -3′
*Mfn1*	5′-AGC TCG GAA TCG GAT CTT TTT-3′	5′ -CTG CTG ACT GCG AGA TAC ACT -3′
*Mfn2*	5′- GCC GGA CGA GCA ATG GGA A-3′	5′ -TCT TCT GAG CCC TCC GTG A -3′
*OPA1*	5′ -ACC CAA AGG AAA GGA ACA CGA -3′	5′- TGA AGT AGA TGG CTG CGT CCC-3′
*Drp1*	5′ -AAG CCC TGA GCC AAT CCA TCT-3′	5′-GAT TAC TGA TGA ACC GAA GAA-3′
*Fis1*	5′ -AAG CCC TGA GCC AAT CCA TCT-3′	5′- GAT TAC TGA TGA ACC GAA GAA -3′
*Caspase1*	5′ -ACA CCC ACT CGT ACA CGT CTT -3′	5′- TTG TCA TCT CCA GAG CTG TGA-3′
*IL-1β*	5′-TGT GGC AGC TAC CTA TGT CTT-3′	5′-AGT GCA GCT GTC TAA TGG GAA-3′
*β-Actin*	5′-GCA GCG GGA TTA TGT CTT CTA-3′	5′-TTT CTT CAT GGC CTT GTC AAT-3′

## Data Availability

The analyzed data are available from the corresponding author on reasonable request.
